The article "Disorder Genes Regulate the Progression of Ischemic Stroke through the NF-κB Signaling Pathway" was retracted in 2024. Reasons: signs of a paper mill; suspected computer-generated content; unreliable results or conclusions; concerns about the data.

# Disorder Genes Regulate the Progression of Ischemic Stroke through the NF-*κ*B Signaling Pathway

**DOI:** 10.1155/2021/2464269

**Published:** 2021-10-27

**Authors:** Wei Wei, Wenqiang Xin, Yufeng Tang, Zhonglun Chen, Yue Heng, Mingjun Pu, Bufan Yang, Jiacai Zuo, Jingfeng Duan

**Affiliations:** ^1^Department of Neurology, Mianyang Central Hospital, Mianyang 621000, China; ^2^Department of Neurosurgery, Tianjin Medical University General Hospital, Tianjin 300052, China

## Abstract

Stroke is an acute cerebrovascular disease, including ischemic and hemorrhagic stroke. Stroke is the second leading cause of death after ischemic heart disease, which accounts for 9% of the global death toll. To explore the molecular mechanisms of the effects of the dysregulated factors, in the GEO database, we obtained transcriptome data from 24 h/72 h of mice with ischemic stroke and 24 h/72 h of normal mice. We then performed differential gene analysis, coexpression analysis, enrichment analysis, and regulator prediction bioinformatics analysis to identify the potential genes. We made a comparison between the ischemic stroke 72 h and the ischemic stroke for 24 h, and 5103 differential genes were obtained (*p* < 0.05). Four functional barrier modules were obtained by weighted gene coexpression network analysis. The critical genes of each module were ASTL, Zfp472, Fmr1 gene, and Nap1l1. The results of the enrichment analysis showed ncRNA metabolism, microRNAs in cancer, and biosynthesis of amino acids. These three functions and pathways have the most considerable count value. The regulators of the regulatory dysfunction module were predicted by pivotal analysis of TF and noncoding RNA, and critical regulators including NFKB1 (NF-*κ*B1), NFKBIA, CTNNB1, and SP1 were obtained. Finally, the pivotal target gene found that CTNNB1, NFKB1, NFKBia, and Sp1 are involved in 18, 32, 2, and 60 target genes, respectively. Therefore, we believe that NFKB1 and Sp1 have a potential role in the progression of ischemic stroke. The NFKB signaling pathway promotes inflammatory cytokines and regulates the progression of ischemic stroke.

## 1. Introduction

Ischemic stroke is the second leading cause of death after ischemic heart disease, accounting for 9% of the global death toll. According to the World Health Organization, 15 million people worldwide suffer from stroke each year, of which more than 6 million die and another 5 million are permanently disabled. Evidence suggests that after ischemic stroke, ROS production rapidly increases overwhelming antioxidant defenses, causing further tissue damage [1].

According to statistics, there are about 25.7 million stroke survivors in the world, and ischemic stroke is still the most common type of stroke. Risk factors include hypertension, hyperlipidemia, and atrial fibrillation as well as bad habits [2]. Ischemic stroke is a multifactorial disease that causes a severe burden of noncommunicable diseases in developing countries. Diabetes, obesity, high blood pressure, and heart disease are prone to ischemic stroke, and the incidence of ischemic stroke is also proportional to body weight. It is mainly because the brain is the tissue that stores energy and it is an active endocrine organ that secretes many humoral factors [3]. Cerebral ischemia activates a cascade of multiple cell type-specific pathological mechanisms. In the central nervous system, ischemic stroke is caused by ischemia that consists of platelets, endothelial cells, and neutrophils. Damage to cell diversity after ischemia can induce cell death or tissue damage in the brain. According to this principle, studies have been conducted to block ASK1 by pharmacological and genetic manipulation to enhance neuroprotection. It thus prevents ischemic stroke [4]. Some studies suggest that blood-brain barrier protection can be used as a treatment strategy for ischemic stroke. The blood-brain barrier (BBB) is an essential component of the neurovascular unit (NVU), which contains tight junction (TJ) proteins, nutrient transporters, and various ions to maintain healthy brain physiology. The destruction of BBB is the primary pathological marker in the process of ischemic stroke [5], which will regulate matrix metalloproteinases and inflammatory regulators after stimulation. Recent studies have found that ischemic stroke is also associated with lipoprotein A (LPA). It has the potential to cause arteriosclerosis, but there are conflicts in gender-related risk differences [6]. Further studies have also shown that ischemic stroke weight aortic stiffness is also associated with AHR.

In ischemic stroke, studies suggest that the underlying pathophysiological mechanism is impaired baroreceptor function in rigid arteries, leading to impaired BP self-regulation [7]. The study also believes that high heart rate is a strong predictor of poor prognosis in patients with ischemic stroke and can be used to improve their prognosis [8]. A large number of studies have shown that the main progress of ischemic stroke is related to proinflammatory cytokines, including plasma tumor necrosis factor-*α* (TNF-*α*) and interleukin (IL-1*β*, IL-6, IL-8, IL-10, and IL-17). The levels of proinflammatory cytokines were determined by enzyme-linked immunosorbent assay (ELISA). The National Institutes of Health Stroke Scale (NIHSS) can also be used to assess the severity of stroke in patients with ischemic stroke. The results indicate that the severity of the disease is associated with increased inflammation [9]. Currently, the drugs for the treatment of ischemic stroke are perillyl alcohol (PA), probenecid, minocycline, and shikonin. Perillo (PA) has antioxidant and anti-inflammatory properties that protect the nerve by mitigating oxidative stress and inflammation [10]. Probenecid is a potent pannexin 1-channel inhibitor that prevents ischemic brain damage by inhibiting brain inflammation and edema [11, 12]. Minocycline can alleviate the glial cell production of proinflammatory cytokines on neural stem cells [13]. Shikonin effectively protects the brain from damage by regulating the inflammatory response and improving BBB permeability [14]. Studies have shown that embryonic stem cells, induced pluripotent stem cells, neural stem cells, and mesenchymal stem cells may be beneficial for cell replacement and beneficial for neuroprotection, regulating inflammation and immune response [15]. The purpose of this study was to understand the mechanism of proinflammatory cytokines in the regulation of ischemic stroke and provide a reference for the clinical treatment of ischemic stroke.

## 2. Materials and Methods

### 2.1. Data Resource

All data in this study were from GEO, the microarray data of the database numbered GSE102558 was selected, and the data of the probe in the experiment was GPL20710. In this dataset, induced ischemic stroke (middle cerebral artery occlusion) in wild-type animals was applied. After 24 and 72 hours, the isolated cardiac RNA were extracted. For both time points, we generated and analyzed sham operated control animals. The Gene Expressions Comprehensive Database is an international public knowledge base. With advances in bioinformatics, GEO can now accept high-throughput sequencing data for other data applications, including detection of genomic methylation, chromosome structure, and genomic and proteome interactions. We downloaded the transcriptome data of cardiac samples of 24 h/72 h ischemic stroke mice (6 each) and 24 h/72 h normal mice (6 each) in GEO for differential analysis of gene differential expression [16].

### 2.2. Difference Analysis

We analyzed the processing of the GEO specimens and the sample microarray data obtained in the R language. The difference analysis of the gene expression map data in this study is mainly realized by using the R language limma package [17–19], which contains preliminary screening and correction of data. We used the correct background function to calibrate and standardize the data, setting the threshold of *p* < 0.05 and ∣logFC | >2, which is exceptionally significant. We then used the quantile normalization method in the normalizeBetweenArrays function to filter out the control probes in the GPL20710 data and the low-expressed probes. We used the eBayes and lmfit functions to identify differentially expressed genes in the dataset, with default parameters.

### 2.3. Coexpression Analysis

To explore the molecular mechanisms of gene expression during the progression of ischemic stroke, we performed a differential analysis between 24 h/72 h (6 each) of ischemic stroke mice and 24 h/72 h (6 each) of normal mice. Thus, the expression profile of the differential gene was made based on the obtained 5103 differential genes. We used a weighted gene coexpression network analysis (WGCNA) [20] to analyze the differential expression profile matrix obtained from the study. The aim is to explore the synergistic expression of differential genes, thereby clustering to form gene modules with the same/similar expression function, which we also call functional disorder modules. We used the correlation coefficient weighting method to take the *N*-th power of the correlation coefficient between genes and then obtained the correlation coefficient between any two genes. Before the results of the correlation coefficients were clustered, the links between the genes in the network need to be subject to the scale-free network distribution to be more biologically significant. After obtaining the weighted correlation coefficients, we clustered them and constructed a clustering tree by correlation coefficients between different genes. The different branches of the cluster tree represented different functional barrier modules. Contrasting colors represented different modules, and there was a high correlation between the genes in the same branch. Based on the ability of the gene to regulate in each dysfunction module, we unearthed the essential genes that cause the dysfunction of the functional modules.

### 2.4. Enrichment Analysis

After obtaining the functional disorder module, it is necessary to understand the function and signaling pathway of the critical genes involved in the module, in order to better understand the molecular mechanism of ischemic stroke healing. The enrichment analysis of the function and pathway of the gene of the dysfunctional module is an effective means to explore the potential mechanism of gene expression of ischemic stroke healing for myocarditis. In this study, we took acute wound specimens and samples on the third postoperative day.

On the 3rd and seventh day after surgery, we obtained 14 functional disorder modules by coexpression analysis. We used the Bioconductor's clusterProfiler package [21] in the R language for enrichment analysis of functions and pathways. With the clusterProfiler package, we can perform statistical analysis and visualization of functional clustering of genes or gene clusters.

GlueGO was used to enrich the functions and paths of each module and build a corresponding function and access network. We identified modules that participate in the ratio of corresponding functions and pathways to find the highest channel. In this study, the function of participating in neutrophils and vesicles was found to have a higher count value.

### 2.5. Regulator Analysis

Gene transcription and posttranscriptional regulation are often centered on noncoding RNA (ncRNA) and transcription factor (TF). Therefore, we also believe that ncRNA and TF are regulators of the entire molecular mechanism, so we need to analyze its regulators to understand the molecular mechanism of ischemic stroke healing better. We scientifically predict and test the role of dysfunction modules for skin posthealing by bioinformatics, thereby improving the accuracy and efficiency of the experiment. During the ncRNA pivot analysis, we screened the control lines between each regulator and each module to be greater than or equal to 6 plots, and for the significance of the abdominal muscle targets between each module, *p* value < 0.01. In the course of TF pivot analysis, we calculated the target significance of enrichment in each module based on the hypergeometric test (*p* value < 0.01). The data is finally entered into Cytoscape to make a pivot-module network diagram.

### 2.6. Back to Target Genes

Based on the obtained ncRNA and TF that drive ischemic stroke, the target genes are traced back. A single regulator can involve several target genes. We used the interaction pairs in the raid database to backtrack the obtained ncRNA and TF. The interactions between humans and mice were screened separately, and then, score > 0.5 was selected for combined deduplication. We finally obtained ncRNA and TF target genes.

## 3. Results

### 3.1. Determining the Expression of Dysregulated Molecules in Ischemic Stroke

We performed differential gene analysis by comparing transcriptome data from cardiac samples. A broad threshold *p* < 0.05 was set, and 5103 differential genes were obtained (Table S1). Among the differential genes, we believe that there are expression disorders that regulate the progression of ischemic stroke.

### 3.2. Identify Ischemic Stroke-Related Functional Disorder Modules

Biological networks can characterize the underlying pathogenic mechanisms of biological disease and clusters form modules, each of which characterizes a potential mechanism of action. Each module also contains the core genes for its function, and core genetic disorders will drive the module to dysregulate, causing abnormalities in a global function, leading to disease. In order to study the functional disorder module related to the progression of ischemic stroke, it is necessary to construct the expression profile matrix in the sample for the above 5103 differential genes and their interaction genes. Based on the weighted gene coexpression network analysis (WGCNA), we observed that these genes showed significant grouping expression in the samples, and the genes with similar behavioral expression formed a module for coexpression clustering. In this study, we aggregated gene expression behavior into modules. It helps us to observe the complex collaborative relationships between these genes from the perspective of expression behavior. Among the four functional disorder modules (Figures 1(a) and 1(b)), based on the functional disorder module, we further identified the essential genes of each module and obtained the four core genes Astl, Zfp472, Fmr1, and Napl1l1 (Table 1). We associated the module with the phenotype data and plotted it (Figure 1(c)). In the sample, the turquoise module was associated with gene expression 24 h of ischemic stroke. In the 72 h sample of ischemic stroke, MEblue, MEbrown, and yellow were associated with gene expression 72 h of ischemic stroke.

### 3.3. Functions and Pathways Involved in the Gene of Interest

Function and pathway are essential mediators of the physiological response of the disease. We performed functional and pathway enrichment analysis on the four functional barrier modules and obtained a total of 22056 biological processes, 2693 cells, 4840 molecular functions, and 993 KEGG pathways (Table S2). The highest function of count is ribosomal large subunit assembly, and the highest path of count is steroid biosynthesis. We extracted some of the functions and pathways of interest from the table for analysis and bubble diagrams (Figures 2(a) and 2(b)). The results showed that the ncRNA metabolic process, microRNAs in cancer, and biosynthesis of amino acids had the most substantial count value. From the figure, we can see that ncRNA and miRNA are related to the whole process of ischemic stroke, mainly to regulate the biosynthesis of amino acids and affect the expression of proteins and the proinflammatory cytokines. The endogenous polypeptide produced by the immune system cells with many powerful biological effects can mediate a variety of immune responses. Therefore, we believe that critical genes mainly affect the progression of ischemic stroke by regulating the production of proinflammatory cytokines.

### 3.4. ncRNA and TF That Drive the Development of Ischemic Stroke

Through the above analysis, we obtained functional and critical genes that are associated with the progression of ischemic stroke. From the perspective of systems biology and systems genetics, transcription and posttranscriptional regulation of genes have long been recognized as a critical regulator of disease development and progression. Transcription factors and ncRNA are conventional regulators. We performed a pivotal analysis of coexpressed modular genes to explore critical transcriptional regulators in the progression of ischemic stroke. Pivot analysis was performed based on the targeted regulation of the TF and ncRNA on the module gene, and a network diagram of the relationship between TF and ncRNA was obtained (Figures 3(a) and 3(b)). The results showed a total of 53 ncRNAs involving 56 ncRNA-module pairs. There are 17 TFs involving 19 TF-module pairs (Tables S3 and S4). In the ncRNA pivot assay, miR-10b-5p was most ligated to ncRNA. In the analysis, the modules and TF connections are more NFKB1, Ctnnb1. NFKB1 has shown its pivotal role in the analysis of the functions and pathways in which our genes of interest are involved. Therefore, we believe that NFKB1 has a potential regulatory role in the progression of ischemic stroke. The mechanism of action may be that proinflammatory cytokines regulate the progression of ischemic stroke through the NFKB signaling pathway.

### 3.5. Backtracking the Target Gene of the Pivot

After analyzing the ncRNA and TF that drive ischemic stroke, we obtained a network diagram of their interactions. The ncRNA or TF-related target genes are not represented in the network diagram, so we need to backtrack the obtained ncRNA pivot and TF pivot (Tables S5 and S6). The results of retrospective target genes showed that G730013B05Rik and mmu-miR-362-3p involved 103 and 92 target genes, respectively, and Ctnnb1, NFKB1, NFKBia, and Sp1 involved 18, 32, 2, and 60 target genes, respectively. Therefore, we believe that G730013B05Rik, mmu-miR-362-3p, NFKB1, and Sp1 have potential roles in the progression of ischemic stroke. The mechanism of action may be that proinflammatory cytokines regulate the progression of ischemic stroke through the NFKB signaling pathway.

## 4. Discussion

Ischemic stroke is considered to be one of the major health problems in the world with high mortality and morbidity. Studies have found that it is associated with inflammation, oxidative stress, and excitotoxicity. Ischemic stroke is often required to be treated in a short period, so it is needed to developing a more effective neuroprotective agent in the direction of treatment. For targeted treatment and prevention of ischemic stroke, we need to understand the mechanisms of dysfunction. Recent studies have shown that both endogenous basic fibroblast growth factor (bFGF), apolipoprotein E gene (APOE), BET 2, and remote ischemic preconditioning (RIPerC) are significantly reduced with ischemic related to stroke. bFGF is not only related to neuroprotection and neurotrophic effects but also excessive astrocyte proliferation and glial scar formation after neuronal injury. The presence of the E4 allele is a risk factor for ischemic cerebrovascular disease. RIPerC prevents collateral collapse from having neuroprotective effects [22–25]. In order to study its mechanism of action, we need to analyze its differential genes. We collected transcriptome data from 24 h/72 h in ischemic stroke mice and 24 h/72 h in normal mice (GSE102558). Difference analysis and coexpression analysis were performed after standardization [26]. After WGCNA coexpression network analysis, a total of 5103 differential genes were obtained. Due to a large number of differential genes, we need to further cluster these differential genes. We clustered similarly expressed genes to obtain four related functional disorder modules, including the four core genes Astl, Zfp472, Fmr1, and Nap1l1. Also, other studies have shown that single-nucleotide polymorphisms (SNPs) are associated with ischemic stroke, mainly affected by ZNF208 and HNF1A [27, 28]. ADAMTS-4 has an anti-inflammatory effect mainly in the CNS. There are more and more studies on promoting ischemic stroke [29, 30], but we still need to continue to analyze how proinflammatory cytokines work. We analyzed the functions and pathways involved in differential genes, and the highest function of count was ribosomal large subunit assembly, and the highest path of count was steroid biosynthesis. Analysis of the functions and pathways of interest revealed that the larger count values were mainly focused on the regulation of amino acid biosynthesis. Proinflammatory cytokines are endogenous polypeptides produced by the immune system cells with many powerful biological effects. Therefore, we believe that the gene of interest mainly affects the progression of ischemic stroke by regulating the production of proinflammatory cytokines. The main proinflammatory cytokines in the study were tumor necrosis factor alpha (TNF-alpha) and interleukins. Studies on TNF-alpha have shown that the immune system can affect brain function quickly and adversely. TNF-*α* signaling may be a target of neuroprotection, which may be involved in the pathogenesis of ischemic stroke [30, 31]. Interleukins are also typical proinflammatory cytokines, and the level of interleukins after ischemia is increased [32–34], suggesting a potential mechanism of action with ischemic stroke. It is noteworthy that studies have shown that IL-6, IL-1*β*, and TNF*α* are both inhibited by TLR4/NF-*κ*B [35]. In this study, the ncRNA and TF were analyzed by pivotal analysis. The module and TF were more connected with NFKB1. The NF-*κ*B signaling pathway acts as a “molecular switch” in ischemic stroke. When it is on, numerous proinflammatory cytokines, cellular adhesion molecules, and immunologic mediators are expressed or synthesized and secreted, promoting an inflammatory response. Studies have shown that NFKB1 (NF-*κ*B1) is significantly involved in the progression of ischemic stroke. We have learned that NFKB1 (NF-*κ*B1) can be cotranslated by the 26S proteasome to produce 105KD protein. Proinflammatory cytokines are precisely peptides, so we believe that the mechanism of action may be that proinflammatory cytokines regulate the progression of ischemic stroke through the NFKB signaling pathway. Comparing the studies done by other scholars, we found that the genes of the NFKB family do significantly regulate the progression of ischemic stroke. The TLR4/MyD88/NF-*κ*B signaling pathway and the ROS/TLR4/NF-*κ*B inflammatory signaling pathway [36, 37] have all shown their regulatory mechanisms. Proinflammatory and anti-inflammatory effects, as well as neuroprotection, are associated with the NF-*κ*B signaling pathway [38, 39]. However, the major limitation is there is no further experimental validation for our results, which will be performed soon. In summary, the study suggests that the NFKB signaling pathway mainly regulates the role of proinflammatory cytokines in ischemic stroke.

## Figures and Tables

**Figure 1:** Synergistic expression of differential genes between acute wound specimens and postoperative wounds on days 3 and 7. (a) The 14 coexpression panels obtained by clustering were identified as modules, and 14 colors represent 14 coexpression modules. (b) Expression heat map of all genes in the sample, whose expression behavior is clustered into 14 coexpression modules. (c) Each row represents a module, each column represents a phenotype, the color of each cell is mapped by the corresponding correlation coefficient, the value is from -1 to 1, the color transitions from blue to white, and then transitions to red.

**Figure 2:** Functional and pathway enrichment analysis excerpts of the module gene. (a) Module gene GO function enrichment analysis excerpt. The color increases from blue to purple, and the enrichment increases significantly. The larger the circle, the more significant the proportion of the gene in the module that accounts for the GO function. (b) Module gene KEGG pathway enrichment analysis excerpt. The color increases from blue to purple, and the enrichment increases significantly. The larger the circle, the more significant the proportion of the gene in the KEGG pathway entry.

**Figure 3:** Regulatory effect of the regulator on the dysfunction module. (a) Orange circles represent modules and yellow circles represent ncRNA. (b) The green circle represents the module, and the purple circle represents the TF.

**Table 1:** Hub gene of modules.

Color	Hudgens	Module
Blue	Astl	m4
Brown	Zfp472	m3
Turquoise	Fmr1	m1
Yellow	Nap1l1	m2

## Data Availability

The datasets used and/or analyzed during the present study are available from the corresponding author on reasonable request.

## Supplementary Materials

Supplementary 1 Table S1: DEG of genes (*p* value < 0.05).

Supplementary 2 Table S2: enrichment_all.

Supplementary 3 Table S3: ncRNA pivot that regulates modular genes.

Supplementary 4 Table S4: TF pivot that regulates modular genes.

Supplementary 5 Table S5: ncRNA_target_gene.

Supplementary 6 Table S6: TF_target_gene.
